The article "Multiclass Classification for Detection of COVID-19 Infection in Chest X-Rays Using CNN" was published in 2022. Journal: Comput Intell Neurosci.

# Multiclass Classification for Detection of COVID-19 Infection in Chest X-Rays Using CNN

**DOI:** 10.1155/2022/3289809

**Published:** 2022-08-11

**Authors:** Rawan Saqer Alharbi, Hadeel Aysan Alsaadi, S. Manimurugan, T. Anitha, Minilu Dejene

**Affiliations:** ^1^Department of Artificial Intelligence, Industrial Innovation & Robotics Center, Faculty of Computers and Information Technology, University of Tabuk, Tabuk City, Saudi Arabia; ^2^Department of Computer Science and Engineering, Saveetha School of Engineering, Saveetha Institute of Medical and Technical Sciences (Deemed to be University), Chennai, Tamilnadu, India; ^3^Department of Biotechnology, College of Biological and Chemical Engineering, Addis Ababa Science and Technology University, Addis Ababa, Ethiopia

## Abstract

Coronavirus took the world by surprise and caused a lot of trouble in all the important fields in life. The complexity of dealing with coronavirus lies in the fact that it is highly infectious and is a novel virus which is hard to detect with exact precision. The typical detection method for COVID-19 infection is the RT-PCR but it is a rather expensive method which is also invasive and has a high margin of error. Radiographies are a good alternative for COVID-19 detection given the experience of the radiologist and his learning capabilities. To make an accurate detection from chest X-Rays, deep learning technologies can be involved to analyze the radiographs, learn distinctive patterns of coronavirus' presence, find these patterns in the tested radiograph, and determine whether the sample is actually COVID-19 positive or negative. In this study, we propose a model based on deep learning technology using Convolutional Neural Networks and training it on a dataset containing a total of over 35,000 chest X-Ray images, nearly 16,000 for COVID-19 positive images, 15,000 for normal images, and 5,000 for pneumonia-positive images. The model's performance was assessed in terms of accuracy, precision, recall, and *F*1-score, and it achieved 99% accuracy, 0.98 precision, 1.02 recall, and 99.0% *F*1-score, thus outperforming other deep learning models from other studies.

## 1. Introduction

Nowadays, research on the healthcare domain holds a great importance and is a key player in refining the living standards of people all over the globe. This importance reveals itself by discussing the successful diagnosis procedures as well as identifying the more accurate diagnosis tools for patients. Medical professionals face several challenges in their practice, and therefore healthcare research affects the doctor or practitioner as much as it affects the patient in terms of steering away from inaccurate diagnosis leading to unnecessary medication or other kind of treatment [1].

The article "Multiclass Classification for Detection of COVID-19 Infection in Chest X-Rays Using CNN" was published in 2022. Journal: Comput Intell Neurosci.

Computer systems can produce accurate results rapidly if relied on novel technologies for image processing [2]. Among the many available technologies, deep learning stands out as the technology of choice for processing images, including radiographs. Introducing deep learning models in the biomedical field has benefitted this area such that several deep learning models are frequently implemented to create automated systems for the detection of diverse diseases [3]. A sub-branch of deep learning, known as Convolution Neural Network (CNN), is strongly present in the image processing domain. CNN also established itself in the field of medical diagnosis among various other areas [4]. Typically, with the recent major worldwide health crisis, deep learning and CNNs specifically were targeted towards research about COVID-19 and its proper detection.

As it became well known, the discovery of the new coronavirus took place in late-2019 in China, in the city of Wuhan, where people were suffering from a lung infection, otherwise described as pneumonia, from an unknown source [5]. This mysterious infection was extremely contagious and managed to travel through the entire China and shortly to the entire world in a remarkably short period of time. This new infection was soon found to be from a viral source, previously known to humans, which gained new stronger capabilities, where the virus acquired the name “SARS-CoV-2” whereas the disease was termed COVID-19. From its early emergence, the novel coronavirus had public health authorities worried and was labeled an “emergency” before being officially declared in January 2020 as a pandemic [6].

Coronavirus disease is highly infectious and causes an array of symptoms that vary between being mild or even having no symptoms at all to extreme cases that could ultimately lead to death. Coronavirus infection is concentrated in the organs of the respiratory tract especially the lungs. COVID-19 symptoms are commonly a high fever, general fatigue, dry coughs, headaches, dyspnea, organ failure such as kidneys or liver, and overall respiratory illness. In more severe cases, COVID-19 patients are hospitalized and must be given extensive care to prevent death. In fact, until January 2022, the World Health Organization recorded over 334 million cases of corona infections worldwide, with over 5 million deaths [7]. These statistics clearly reflect the impact of the coronavirus spread on public health in all countries without exceptions. Moreover, the coronavirus has acquired high adaptability especially when this is coupled with factors such as the immune system of the hosts, the medical interventions, and the environmental factors. These factors lead the virus to accumulate genetic mutations and evolve, creating new strains and variants that have also caused outbreaks in several countries [8]. These mutations affect the capabilities of the new variant strains of coronavirus, making them spread even faster than the initial strain (alpha), and have different symptoms from each other. The Delta variant of the coronavirus (B.1.617.2) is spreading faster and is leading to even more infections among the populations. In addition, the Omicron variant (B.1.1.529) has also emerged and is causing even more trouble in the public health area, especially because these new strains seem to be immune to the existing COVID-19 vaccines [9] shown in Figure 1.

The article "Multiclass Classification for Detection of COVID-19 Infection in Chest X-Rays Using CNN" was published in 2022. Journal: Comput Intell Neurosci.

Identifying coronavirus infection is extremely important since asymptomatic carriers of the virus can go on and spread the virus even without knowing that they carry it. The typical detection method for corona infection is through RNA-based assay using nasopharyngeal swabs, otherwise known as RT-PCR. Unfortunately, this kind of identification test is invasive to the patient and uncomfortable and consumes a lot of time, in addition to having an overall shortage of swabs, reagents, and transfer media. Added to that the fact that PCR tests are not 100% accurate, rather there is a significant percentage of tests that come out as false negative. This kind of result also affects the spread of the virus and thus needs controlling [10]. Yet other methods can be utilized for identification of COVID-19 infections through chest X-Ray scans. Chest X-Ray scans fall among the least expensive tests and produce results almost immediately. X-Rays can be especially important in corona detection because they can be performed in isolated areas to prevent any further spread of the virus [10].

Using computer-generated images for the detection of corona viral infection in the lungs has many benefits and many challenges. The challenge is that radiographs require skilled radiologists that are informed enough to be able to identify the distinctive features that the coronavirus creates within the lungs. Furthermore, the chest X-Ray images for the naked eye can show no presence of the infection simply because the virus has not affected the lungs severely yet. Therefore, using chest X-Rays, for example, for corona infection detection is not 100% accurate, unless it was in parallel with the traditional PCR test [11]. On the other hand, there are several benefits of using computer images which include (1) fast triaging, which classifies patients according to priority with respect to their extent of infection, since X-Rays can determine the severity of the infection on lungs; (2) accessibility, ease of use, and being patient-friendly (not invasive), and (3) flexibility, since it does not require direct contact between the patient and the medical staff [12].

The article "Multiclass Classification for Detection of COVID-19 Infection in Chest X-Rays Using CNN" was published in 2022. Journal: Comput Intell Neurosci.

Corona viral infection can be mistaken with viral pneumonia infection, since a person infected with pneumonia can have an array of symptoms ranging from being mild, to being extremely uncomfortable, and he/she might even need urgent medical attention. Coughing, exhibiting hyperthermia, sweating or shivering, losing appetite, and experiencing fast heartbeats are among the most common symptoms of pneumonia infection. However, in more serious cases, an infected individual might cough up blood and have difficulty in breathing or faint [13]. By definition, pneumonia is the medical condition in which one or both lungs get filled with fluids or pus, which makes the respiration process troublesome [14]. Pneumonia is accountable for more than 500 thousand emergency room attendances yearly. Pneumonia is predominant in adults. Nonetheless, it poses as the primary cause of death in children below 5 years among all the infectious diseases. Approximately, pneumonia kills around 2,400 children per day [15]. There exist several criteria by which pneumonia can be classified such as the origin of infection whether it is hospital-acquired or community acquired, the host factor and its respective immunity, and the causative pathogen [16]. Classifying pneumonia according to the causative pathogen allows the grouping of the medical condition into bacterial pneumonia which is triggered by bacterial proliferation, viral pneumonia produced by a viral infection, and fungal pneumonia which is the result of fungal infections [17].

In fact, the continuously evolving technology can benefit the medical field by detecting coronavirus and pneumonia through analyzing chest X-Rays. Artificial intelligence for one is often used in medical image processing shown in Figure 2. Successful machine learning techniques can lead to faster assessment of chest X-Ray images and thus help the radiologists to screen potential patients in a shorter period of time. Studies using deep neural networks have shown the effectiveness of the method in the diagnosis of pneumonia [9]. Artificial intelligence can actually have a great impact in all fields of medical fields such as diagnosis, survillance, delivery, service automation, and recovery monitoring are illustrated in Figure 2 below.

Two main fields of artificial intelligence, namely, the deep learning and machine learning approaches played an important role in the detection of COVID-19 positive patients. The deep learning techniques acquire knowledge of the hierarchal feature learning which makes them strong in learning the most complicated features with ease. In the cases of corona infection, some patterns such as GGo, pleural effusion, consolidation among others appear. These patterns can also be identified in pneumonia cases which makes it tricky. However, deep learning technology can learn the very exact patterns created by COVID-19 infections and thus be able to distinguish them in radiographs. Actually, studies show that using deep learning in such identification tasks provides high specificity and sensitivity and ultimately high accuracy. This comes along with low rates of false identification, whether it is the false negative or false positive. This way, artificial intelligence approaches are viewed as robust, accurate, and economical [15]. Neural networks for instance are widely used nowadays in medical applications because of their flexibility and ability to handle nonlinear systems.

The article "Multiclass Classification for Detection of COVID-19 Infection in Chest X-Rays Using CNN" was published in 2022. Journal: Comput Intell Neurosci.

After conducting several studies, it became clear that CNN can be sued to extract various patterns and features without the need for preprocessing. This is possible due to factors such as the use of replicated layers and shared weights, which cause the learning process of a CNN model to be a lot easier. In addition, far-reaching studies on CNN allowed the creation of several varying architectures based on CNN such as Lenet, Faster R-CNN, ResNet, and VGGs [16, 18, 19].

The layering of a convolutional neural network consists of an arrangement or stacking of many trainable steps that are usually followed by a classifier module responsible for segregation of different features per input and output [20]. As an input, CNNs accept videos, images, or audio. In the case of colored images, the input consists of 2D array of colors, and the output is a collection of the extracted features one by one in order to create a feature map. The process of network training includes feeding the input, followed by computations, and producing an output. The final output must be compared with labeled data which show the correct answer and the result of the network.

When a patient goes for a chest X-Rays, the results are given to him in a form of image. The same image on the computer can be used to analyze it and extract the features from it by using CNN models. As a matter of fact, there exist several studies that employ CNN models to identify the presence of pneumonia infection, as well as COVID-19 infections. Such models are the VGGs (16 and 19), ResNet, Xception, and DenseNet [21]. These models are either developed from scratch or modified and fine-tuned in order to produce accurate results for the detection of COVID-19 infections in lung X-Rays. Several studies were done on applying deep learning and CNNs in particular, to identify the infection of patients with coronavirus or with viral pneumonia.

The article "Multiclass Classification for Detection of COVID-19 Infection in Chest X-Rays Using CNN" was published in 2022. Journal: Comput Intell Neurosci.

In this study, we focus on creating an enhanced model capable of accurately distinguishing between the COVID-19 infection and the viral pneumonia infection through analyzing and classifying chest X-Ray images. The study trains the model on a large dataset and implements a CNN architecture to properly classify the images.

## 2. Related Works

The majority of the previous studies of course was focused on the detection of pneumonia as it is a health risk of a significant impact. Even after the breakout of coronavirus and its widespread, research continues to be done on pneumonia and its classification, especially stressing its origin because the origin of pneumonia can greatly impact the healing process due to the proper medication. New research papers still emerge discussing the application of machine learning in pneumonia detection. After the corona pandemic, research was also directed towards finding machine learning applications to detect and identify the coronavirus infection in a quick and non-invasive way. For this reason, several studies focus on discriminating COVID-19 infections from non-COVID-19 infections.

The paper by Panwar et al. [22] discussed the development of a method for rapid detection of COVID-19 in chest X-Ray images through a deep learning technique relying specifically on neural networks, termed nCOVnet. In their paper, the authors aim to distinguish between COVID-19 infected lung images and normal or healthy lung images. The developed dataset is a collection of COVID-19 positive X-Ray images (337 posterior-anterior images) in addition to healthy images from the Kaggle dataset (142 selected images). These images were subjected to preprocessing by applying to resize, RGB, reordering, and data augmentation. The data were carefully split into 70% for training and 30% for testing while making sure there is no data leakage. The data were fed into a model consisting of a pretrained VGG-16 on ImageNet through transfer learning and ReLU and maxpooling layers. The developed algorithm relies on the top layers of the VGG-16 for feature extraction in addition to head layers consisting of five custom trained layers which is capable of shifting the weights forward and backward during iterations. As a result, the model was able to identify COVID-19 in truly infected persons with an error of 2.38%, where the sensitivity is 97.62% and the specificity is 78.57%. The prediction of the positively infected cases had a 97.97% confidence, whereas the confidence in predicting non-COVID cases was 98.68% and both are high values. Overall, the accuracy of the model was calculated to be 88.10%, and the ROC which also reflects the accuracy was 0.88095, which indicated a high accuracy level given the small size of the training dataset.

The article "Multiclass Classification for Detection of COVID-19 Infection in Chest X-Rays Using CNN" was published in 2022. Journal: Comput Intell Neurosci.

Another study aimed at identifying COVID-19 cases from the chest X-Ray images is the study by Khan et al. [20]. The study discusses implementing a model that is based on split-transform-merge concept in addition to region and edge-based extraction of features “STM-RENet.” The model was trained and tested on three different datasets that differ in their content: one dataset contains 6K images of COVID-19 vs. healthy CXR, the second comprises 10K images of COVID-19 vs. other viral infections, and the third is augmented based on the 10K dataset to reach 15K images of COVID-19 vs. other viral infections. A ratio of 8 to 2 was chosen for training and testing, respectively, where the images were also resized and preprocessed. Furthermore, the authors studied the effect of channel boosting (CB) on enhancing the performance of their developed model, where fine-tuned CNNs that are the result of transfer learning are used into the model. Ultimately, the system would start by image input, followed by data augmentation and preprocessing where necessary; then, one of these three models is employed: STM-RENet, CB-STM-RENet, or existing CNN models, in order to distinguish between COVID-19 and non-COVID lung infections. The channel boosted model was shown to have good learning plots that demonstrate its fast learning. In all of the three datasets, CB-STM-RENet performed better than STM-RENet in terms of accuracy, *F*1-score, specificity, sensitivity, and so on. The highest accuracy level recorded by the model is 98.53% in the first dataset and 96.53% in the third dataset which is an imbalanced dataset. Additionally, the model outperformed the previously existing CNN models.

On the other hand, numerous studies merged the two different concepts and were focused on distinguishing between pneumonia infection and COVID-19 infection since that can be a challenging task for radiologists. The study by Khan et al. [21] discussed the capability of different deep learning models in different training techniques in the proper differentiation between COVID-19 infection and viral pneumonia infection. The authors tried to gather a large dataset of chest X-Ray images from several sources such as Kaggle, RSNA, GitHub, and others, which comprise images of COVID-19 patients, normal patients, patients with lung opacity, and pneumonia patients. Therefore, the aim of the study was to perform multiclass classification. Of course, data balancing and augmentation was done on the images that belong to the nonhealthy patients. Next, the features must be extracted from the images, before they are classified, using one of the three pretrained extractors: NasNetMobile, EfficientNetB1, and MobileNetV2. These initial layers are capable of capturing contours and edges from the images and are previously trained on the large dataset ImageNet to gain knowledge through the transfer learning process. Yet, to ensure the most convenient performance of the model, they must be fine-tuned through removing the original classification heads and adding new layers which are the Dense Layers 1 (size 256) and 2 (size 4) in addition to Softmax activation and Adam optimizer. The dataset was divided into training (70%), validation (20%), and testing (10%). To gather a more in-depth results from the study, the authors chose two training strategies, one where the models are pretrained and classified without batch normalization, whereas the second strategy occurred by classification with batch normalization and dropout. As a result, EfficientNetB1 obtained the highest accuracies: 92% and 96.13% in Strategy 1 and 2, respectively, outperforming the other models. However, it is still evident that the batch normalization enhanced the performance of the model by training strategy (2) and increasing its accuracy by 4%. The study also concluded that the number of parameters within a model is not directly linked to its performance.

The article "Multiclass Classification for Detection of COVID-19 Infection in Chest X-Rays Using CNN" was published in 2022. Journal: Comput Intell Neurosci.

The study by Chakraborty et al. [22] also focused on the differentiation between COVID-19 cases and pneumonia cases from chest X-Rays using deep learning technology. The study acquired its dataset from Kaggle and GitHub totaling 10,040 CXR images which include pneumonia cases, COVID-19 cases, and normal cases. After the images are input, image preprocessing and segmentation take place such that all the images that are not labeled as one of the mentioned classes are discarded, in addition to normalization and augmentation. Moreover, FC-DenseNet103 semantic segmentation algorithm and pulmonary contour masks are utilized to get segmented regions of the lung from each image. This dataset is divided as follows: 80% for training (with 10% of these for validation) and 20% for testing. In this deep learning model, the architecture is ResNet18 which was subjected to pretraining to make sure that the efficiency becomes better. This model with the addition of multiclass classification layers is used to classify the data into COVID-19, pneumonia, or normal. In total, the model consisted of 46 layers including convolution, hidden, maxpooling, average pooling, and Softmax layers. The model managed to achieve a 96.43% accuracy rate and a 93.68% sensitivity rate.

The article "Multiclass Classification for Detection of COVID-19 Infection in Chest X-Rays Using CNN" was published in 2022. Journal: Comput Intell Neurosci.

The study done by Xu et al. [23] discussed the development of a new model named “MANet” for differentiating between COVID-19 compared to normal patients, tuberculosis patients, and pneumonia patients (viral or bacterial). The study uses a dataset made up by merging three public datasets in order to train and test the model. The approach depends on a two-stage process which includes segmentation of the CXR from the dataset after being preprocessed, and then the classification stage takes place. Segmentation starts by CXR input followed by preprocessing such as resizing and normalization, and then ResUNet is used to segment the X-Ray images focusing on the lung area, followed by postprocessing in order to reach processed masks as a result. The processed masks are input for the classification stage, where four classifiers are used: ResNet34, ResNet50, InceptionV3, and VGG-16, to determine to which class the CXR belongs. In fact, the performance of the classifiers is compared with and without using Mask Attention (MA) technology. The results show that using MA with any model enhances its performance and increases its accuracy, whereas ResNet50 achieved the highest accuracy levels with MA (96.03%) and without MA (95.78%).

The study by Thakur et al. [24] tackled the issue of binary and multiclass classification of COVID-19 infection by creating two different CNN models that can analyze CXR and CT scans to detect COVID-19. To perform this task, the authors relied on two datasets, the dataset for binary classification consisted of a total of 3,877 images of COVID-19 and healthy images (both CXR and CT), whereas the dataset for multiclass contained 6,077 images of COVID-19, pneumonia, and healthy images. The datasets were initially preprocessed, being resized, normalized, shuffled, and grey scale conversion. The overall combination of images makes up 11,095, divided into 6,077 for training and 5,018 for testing. The created CNN model was evaluated by its accuracy, *F*1-score, precision, sensitivity, and so on. For the binary classification between COVID-19 and normal patients, the accuracy was 99.64% and the *F*1-score was 98.82%; for the multiclass classification between pneumonia, COVID-19, and normal, the accuracy was 99.95% and the *F*1-score was 98.23%.

The Table 1 below demonstrates in detail the performance of each of the studies mentioned in the Literature Review section.

## 3. Methodology

### 3.1. Dataset

This study was focused on achieving impactful results in terms of accuracy of detection and precision, which is why the dataset chosen for this study is large. In fact, we collected several images from different datasets and merged them for our model. These individual datasets are acquired from Kaggle termed “COVIDx CXR-3 Dataset” and “Chest X-ray Images (Pneumonia),” in addition to a healthy/normal lungs dataset. As shown in Figure 3, the corona dataset consists of 16,490 COVID-19 positive images, whereas the pneumonia dataset is made up of 5856 pneumonia-positive CXR images, and the normal dataset is composed of approximately 15,000 healthy lung images.

The article "Multiclass Classification for Detection of COVID-19 Infection in Chest X-Rays Using CNN" was published in 2022. Journal: Comput Intell Neurosci.

### 3.2. Image Preprocessing

The obtained dataset is actually a result of some cleaning done by the researchers, where all the images that were present and are not relevant to this study were discarded, and only those that are either pneumonia, COVID-19, or normal were kept. This is a shortcoming of the model since it is almost impossible to have a perfect public dataset (Table 1).

Before beginning to work on the model, the images in the dataset must be prepared to suit the proposed model and algorithms. In our study, the data as images were stored in csv file, where each image is stored, and its corresponding path and label are also stored. In order to have a homogenous dataset, all images were resized to dimensions (64, 64, 3). The data were split such that 80% were used for training and the remaining 20% were for testing.  Figure 4 illustrates an example of the acquired images in our dataset.

## 4. Proposed Model

### 4.1. Convolutional Neural Networks

In the general form of a CNN, there exist three building-block layers: the convolutional layers that are followed by pooling layers and fully connected layers [25–29]. Convolution neural networks rely on convolution for two main reasons which are (1) parameter sharing where the entirety of the image is processed by the feature detectors and (2) sparsity of connections where a single output value is dependent on a small amount of input values shown in Figure 5.

To do convolution, the filter must be overlayed into the output in order to obtain the summation.

The Stride value determines how many cells are going to be shifted in the right direction in order to obtain the next output value in Figure 6.

Padding also is important for many reasons including the determination of the image border and maintaining the widths and heights of the volume of the convolution without being shrunk in Figure 7. The Convolutional Neural Network (CNN) was used as the core of our model in Figure 8. The Keras applications class allows us to import the CNN, and we used six layers of convolution and max-pooling with a SoftMax output layer. As a result, the output layer is utilized as a multiclass classification layer, since we only have three classification classes, COVID-19, normal, and pneumonia.

The article "Multiclass Classification for Detection of COVID-19 Infection in Chest X-Rays Using CNN" was published in 2022. Journal: Comput Intell Neurosci.

## 5. Results

Upon building up the model and after finishing the necessary steps, the model was tried on 80% of the dataset as previously described.  Figure 9 demonstrates the workflow of the proposed model. In Figures 10–12, the model was trained with a batch size of 32 for 20 epochs. The model was capable of reaching a 0.99 accuracy level in distinguishing between the three different classes: normal, COVID-19, and pneumonia. The system was also capable of reaching similar validation and training accuracies after the first 10 epochs.

Figure 12 represents some of the results obtained after activating the proposed model on the given dataset.

### 5.1. Dataset

The performance of any given model can be assessed through following certain criteria. The models are mostly assessed according to precision, recall, and *F*1-score, in addition to the accuracy. Precision is a measure of the proportion of the data points that our model says are relevant actually and are in fact relevant. Precision can be calculated by the following formula:

(1) $$\begin{array}{c} \text{precision}=\frac{\text{true positive}}{\text{true positive}+\text{false positive}}. \end{array}$$

Recall refers to the percentage of total relevant results correctly classified by our model and can be calculated as follows [30]:

(2) $$\begin{array}{c} \text{recall}=\;\frac{\text{true positive}}{\text{true positive}+\text{false negative}}=\frac{\text{true positive}}{\text{total actual positive}}. \end{array}$$

*F*1-score can be interpreted as the weighted average of the precision and recall, where an *F*1-score reaches its best value at 1 and the worst score at 0 [30]. The *F*1-score formula is described as follows [30]:

(3) $$\begin{array}{c} F1-\text{score}=2\times \;\frac{\text{precision }\times \text{recall}}{\text{precision}+\text{recall}}. \end{array}$$

The overall results of our proposed model are gathered in Table 2.

As a matter of fact, in Figures 13 and 14, when comparing our achieved results with those in the literature review, it becomes evident that our developed model performs exceptionally well when taking into consideration the larger dataset and the precise accurate results in Table 3.

## 6. Conclusion

Coronavirus has invaded the entire world and created a lot of stress both emotionally and medically. With the progress of its spread, medical experts developed methods to identify the characteristics of this viral infection. Radiographies are one of the cheap available options that can be used but contains much challenge due to the novelty of the virus and the emergence of newer strains such as the Delta and Omicron strains. Technology can assist radiologists through examining the chest X-Rays with the help of the deep learning techniques. Unfortunately, the similarities between pneumonia infection and COVID-19 infection as can be seen in a chest X-Ray are complicated, so it is essential to find models that can easily distinguish between them, in order to proceed with the necessary medical process.

The article "Multiclass Classification for Detection of COVID-19 Infection in Chest X-Rays Using CNN" was published in 2022. Journal: Comput Intell Neurosci.

In this study, we proposed a deep learning model based on the CNN architecture, which was trained on a large dataset of 35,000 chest X-Ray images. The proposed model was able to achieve a 99% accuracy with a 99.0% *F*1-score, so it can accurately perform the multiclass classification between normal, pneumonia infection, and COVID-19 infection. Through comparison with other studies, it appears that our proposed model achieves better results, especially when taking to consideration the size of the used dataset.

## Figures and Tables

**Figure 1:** Coronavirus variants scientific names and country of origin as well as discovery date [9].

**Figure 2:** Applications of artificial intelligence in the medical field [9].

**Figure 3:** Distribution of the three classes of images in the dataset according to their count.

**Figure 4:** Example of the images acquired from our dataset.

**Figure 5:** How to do convolution.

**Figure 6:** The Stride.

**Figure 7:** The padding.

**Figure 8:** Architecture of our CNN proposed model.

**Figure 9:** The workflow of the proposed model.

**Figure 10:** Training results of our proposed model.

**Figure 11:** Training accuracy.

**Figure 12:** Obtained results of the proposed model in the three different classes.

**Figure 13:** Performance accuracy an *F*1-score of the proposed model.

**Figure 14:** Comparison of accuracy and *F*1-score of our proposed model with models from literature.

**Table 1:** Illustration of similar studies according to the year, classification type, model, dataset, and performance.

Study	Year	Classification	Model	Dataset	Performance
Application of deep learning for fast detection of COVID-19 in X-Rays using nCOVnet [22]	2020	Binary	VGG-16 model with transfer learning	284 total images of COVID-19 and normal CXR	Accuracy: 88.10% Sensitivity: 97.62% Specificity: 78.57%

COVID-19 detection in chest X-Ray images using a new channel boosted CNN [23]	2022	Binary	Channel boosted split-transform-merge with region and edge-based operation	6,000 (COVID-healthy) 10,000 (COVID-viral infection) 15,000 (COVID-viral infection) CXR	Accuracy: 96.53% *F*1-score: 95%

Chest X-Ray classification for the detection of COVID-19 using deep learning techniques [21]	2022	Multiclass	Efficient NetB1 with transfer learning	21,165 CXR of COVID-19, lungopacity, normal, and pneumonia	Accuracy: 96.13% *F*1-score: 97.50% Sensitivity: 9 6.50%

An efficient deep learning model to detect COVID-19 using chest X-Ray images [22]	2022	Multiclass	ResNet18 with transfer learning	10,040 CXR of COVID-19, pneumonia, and normal	Accuracy: 96.43% Sensitivity: 93.68% *F*1-score: 93%

MANet: A two-stage deep learning method for classification of COVID-19 from chest X-Ray images [23]	2021	Multiclass	ResNet50 with mask attention	6,792 CXR of COVID-19, viral pneumonia, bacterial pneumonia, tuberculosis, and normal	Accuracy: 96.03% *F*1-score: 97%

X-Ray and CT-scan-based automated detection and classification of COVID-19 using convolutional neural networks (CNN) [24]	2021	Multiclass	CNN	6,077 CXR and CT of COVID-19, pneumonia, and normal	Accuracy: 98.28% *F*1-score: 98.23%

The article "Multiclass Classification for Detection of COVID-19 Infection in Chest X-Rays Using CNN" was published in 2022. Journal: Comput Intell Neurosci.

**Table 2:** Performance assessment of the proposed model.

Accuracy	*F*1-score	Precision	Recall
**99.0**	0.99	0.98	1.02

**Table 3:** Comparison of performance of our proposed model with models from literature.

Study	Dataset size	Accuracy (%)	*F*1-score
Our proposed model	35,000 CXR	99.0	99.0%
Panwar et al.	284 CXR	88.10	-
Khan et al.	6K, 10K, 15K CXR	96.53	95%
Alfouzan et al.	21,165 CXR	96.13	97.50%
Chakraborty et al.	10,040 CXR	96.43	93%
Xu et al.	6,792 CXR	96.03	97%
Thakur et al.	6,077 CXR	98.28	98.23%

## Data Availability

The datasets used and/or analyzed during the current study are available from the corresponding author on reasonable request.
